The article "Hyperthermia-Induced NDRG2 Upregulation Inhibits the Invasion of Human Hepatocellular Carcinoma via Suppressing ERK1/2 Signaling Pathway" was retracted in 2020. Reasons: duplicated images; original data or images not available; concerns about the data.

# Hyperthermia-Induced NDRG2 Upregulation Inhibits the Invasion of Human Hepatocellular Carcinoma via Suppressing ERK1/2 Signaling Pathway

**DOI:** 10.1371/journal.pone.0061079

**Published:** 2013-04-22

**Authors:** Yan Guo, Ji Ma, Lin Wu, Qianrong Wang, Xia Li, Xiaoming Li, Yuan Zhang, Jian Zhang, Libo Yao, Jing Zhang, Wenchao Liu

**Affiliations:** 1 Department of Oncology, State Key Discipline of Cell Biology, Xijing Hospital, the Fourth Military Medical University, Shaanxi, China; 2 The State Key Laboratory of Cancer Biology, Department of Biochemistry and Molecular Biology, the Fourth Military Medical University, Shaanxi, China; 3 Experiment Teaching Center, School of Basic Medicine, the Fourth Military Medical University, Shaanxi, China; 4 Department of Neurosurgery, Xijing Hospital, the Fourth Military Medical University, Shaanxi, China; The University of Hong Kong, China

## Abstract

Hyperthermia (HT) has been proven to be able to alter the invasion capacity of cancer cells. However, the detailed mechanisms responsible for the anti-metastasis effects of HT have not been elucidated. N-myc downstream-regulated gene 2 (NDRG2), as a member of the NDRG family, has been suggested to be highly responsive to various stresses and is associated with tumor suppression. The present study aimed to investigate the biological role of NDRG2 in the invasion of human hepatocellular carcinoma (HCC) cells exposed to HT. We found that NDRG2 could be induced by HT at 45°C. In addition, NDRG2 overexpression inhibited the expression of matrix metallo proteinases-2 (MMP-2) and MMP-9 as well as the invasion of HCC cells, whereas knockingdown NDRG2 reversed the anti-invasion effect of HT in vivo. Further investigation revealed that the phosphorylation level of ERK1/2, but not that of JNK and p38MAPK, was reduced in NDRG2 overexpressing cells. Moreover, the knockdown of NDRG2 expression resulted in increased cell invasion, which was rescued by treating the HepG2 cells with the ERK1/2 inhibitor PD98059, but not with the p38MAPK inhibitor SB203580 or the JNK inhibitor SP600125. Finally, the synergistic cooperation of HT at 43°C and NDRG2 expression effectively reduced cytotoxicity and promoted the anti-invasion effect of HT at 45°C. Taken together, these data suggest that NDRG2 can be induced by HT and that it mediates the HT-caused inhibition of invasion in HCC cells by suppressing the ERK1/2 signaling pathway. The combined application of constitutive NDRG2 expression with HT may yield an optimized therapeutic benefit.

## Introduction

Hepatocellular carcinoma (HCC) is one of the most frequent malignancies worldwide, accounting for 85% to 90% of primary liver cancers [1], [2]. Conventional treatments of HCC include surgery, chemotherapy, radiation, percutaneous injection of ethanol (PEI) chemotherapy with anthracyclines or combinations of these treatments. Despite advances in therapeutic strategies, patients with HCC have a poor prognosis because of the propensity of HCC to metastasize [3], [4]. Therefore, the inhibition of invasion and metastasis has been the key factor for the successful treatment of HCC.

Hyperthermia, a minimally invasive treatment with few side effects, has recently been used for cancer therapy. A number of clinical and animal experiments have shown that HT exerts therapeutic effects not only by delaying tumor growth but also by inhibiting lymph node metastasis [5], [6], [7]. Nagashima et al. demonstrated that local HT inhibited the lymph node metastasis of hamster oral squamous cell carcinoma [8]. In vitro research has been carried out to understand the underlying mechanism for this effect. Most of these investigations have focused altering metastasis-related genes, such as vascular endothelial growth factor (VEGF) [9], urokinase type plasminogen activator receptor (uPAR) [10] and MMPs [11], [12]. Among MMPs, MMP-2 and MMP-9 are the critical enzymes that are known to degrade surrounding extracellular matrix components, thus resulting in tumor invasion during cancer metastasis [13]. Although some progress has been made in terms of assessing the biological effect of HT, the molecular mechanism that mediates the anti-metastatic effect of HT has not been elucidated.

N-myc downstream-regulated gene 2 (NDRG2) belongs to the NDRG family, a new family of differentiation-related genes that consists of four members: NDRG1, NDRG2, NDRG3 and NDRG4. Previous studies have reported that NDRG family members are associated with multiple cellular processes, such as proliferation, differentiation and stress responses. NDRG2 was first cloned from glioblastoma using polymerase chain reaction-based subtractive hybridization by our laboratory in 1999 [14]. Decreased expression of NDRG2 is found in a number of human cancers, including breast cancer [15], clear cell renal cell carcinoma [16], liver cancer and pancreatic cancer [17]. The ectopic expression of NDRG2 suppresses the proliferation of tumor cells [14], [18], [19]. In addition, accumulated evidence indicates that the absence of NDRG2 expression in a variety of carcinomas contributes to increased tumor metastatic potential via the regulation of MMP-2/MMP-9 production [20], [21], [22]. All of these findings suggest that NDRG2 has tumor suppressor role. In addition, increasingly more efforts have aimed to determine the role of NDRG2 under stress conditions. We previously reported that NDRG2 can be up-regulated following hypoxia or radiation-induced stress [23], [24]. Foletta et al. demonstrated that NDRG2 expression is highly responsive to different stress conditions in skeletal muscle [25]. However, few studies have examined the response of NDRG2 to HT-induced heat stress and the influence of NDRG2 on the anti-metastatic effect of HT in cancer cells.

In the present study, we sought to clarify the biological role of NDRG2 during HCC invasion under HT conditions. We found that NDRG2 expression was upregulated by heat stress. The overexpression of NDRG2 enhanced the anti-invasion effects of HT in the HCC cell line HepG2, whereas the down-regulation of NDRG2 resulted in attenuated the inhibitory effects of HT on invasion of HCC cells in the xenograft mouse model. We also assessed the underlying intracellular signaling pathway and found that the NDRG2-mediated anti-invasion effect of HT occurs via the suppression of ERK1/2 signaling in human HCC cells. Moreover, the overexpression of NDRG2 synergized with HT to inhibit the invasiveness of HepG2 cells while decreasing spontaneous necrosis.

## Materials and Methods

### Cell lines and culture

Human HCC cell lines (HepG2 and Huh7) were obtained from the Chinese Academy of Sciences (Shanghai, China). All cells were grown in Dulbecco's Modified Eagle Medium (DMEM; Gibco BRL, Grand Island, NY, USA) containing 10% fetal bovine serum (FBS; Gibco BRL, Grand Island, NY, USA) and supplemented with 100 U/ml penicillin and 100 µg/ml streptomycin (Invitrogen, Carlsbad, CA, USA) in a humidified atmosphere of 5% CO_2_ at 37°C.

### Hyperthermia treatment

The T-25 flasks or 6-well plates containing cells at approximately 70% confluence were sealed with parafilm and subjected to HT by immersion in a water bath at 37°C, 39°C, 41°C, 43°C and 45°C for 30 min. Cells subjected to the 37°C water bath served as the controls. All temperatures were maintained within ±0.05°C by testing for accuracy with a thermocouple (Fischer Scientific, Pittsburgh, PA). After the HT treatment, the parafilm was removed, and the flasks and plates were returned to a 37°C incubator for a period of time.

### Lentivirus generation and infection

Recombinant lentiviral vectors were constructed with Invitrogen's ViraPower™ Lentiviral System in our laboratory. The cDNAs of human NDRG2 were cloned and subcloned into the vector pLenti6. Short hairpin RNAs (shRNA) against human NDRG2 were designed using a small interfering RNA design program and were then subcloned into the EcoR I/Age I sites of pLKO-TRC vector. The shRNA sequences specific for NDRG2 were as follows: (shNDRG2: forward, 5′-CCGGGAGGACATG CAGGAAATCATTCTCGAGAATGATTTCCTGCATGTCCTCTTTTTG-3′; reverse, 5′-AATTCAAAAAGAGGACATGCAGGAAATCATTCTCGAGAATGATTTCCTGCATGTCCTC-3′). The sequences for the control nonsense shRNA were as follows: (Scramble: forward, 5′-CCGGAAGGTCTTGTCCTCATCAACACTCGAGTGTTG ATGAGGACAAGACCTTTTTTTG-3′; reverse, 5′–AATTCAAAAAAAGGTCTT GTCCTCATCAACACTCGAGTGTTGATGAGGACAAGACCTT-3′). The HEK-293T cells were transfected with the pLenti6-Cherry/NDRG2, pLKO-Scramble/NDRG2-shRNA, PAX2 and PMD2G lentiviral vectors using Lipofectamine 2000 according to the manufacturer's instructions (Invitrogen, Carlsbad, CA, USA). After 48 h, the lentiviral supernatants were collected, filtered (0.45 µm size filter; Millipore,Billerica, MA, USA), and added onto the HepG2 cells in the presence of 2 µg/ml Blasticidin (Sigma-Aldrich,USA) or 1 µg/ml Polybrene (Sigma-Aldrich,USA) for 6 to 8 h. Two rounds of infection were performed. After infection, the cells that survived this treatment were selected for a week before being analyzed for NDRG2 expression by Western blot.

### In vitro tumor cell invasion assay

The invasive capacity of cells was evaluated using the transwell chamber assay. The upper and lower compartments of the chamber were separated with a polycarbonate filter (8-µm pore size) that was coated with 50 µg of reconstituted basement membrane Matrigel (Collaborative Biomedical Products, Bedford, USA). The cells were trypsinized and seeded in the upper chamber at 1×10^5^ cells/well in serum-free medium. Medium supplemented with 10% FBS (used as a chemo-attractant) was placed in the bottom well, and the cells were then incubated for 24 h at 37°C in a humidified 5% CO_2_ atmosphere. After the incubation, the chambers were removed, and invading cells on the bottom side of the membrane were fixed with methanol for 15 min and stained with gentian violet for 10 min. Invasion was assessed by counting cells in five microscopic fields per well at 400×magnification. The data are representative of triplicate experiments.

### Western blot analysis

Following treatment, cells were harvested and washed in PBS. The cells were homogenized in RIPA lysis buffer (50 mM Tris, pH 7.5, 150 mM NaCl, 1% NP-40, 0.5% sodium deoxycholate, 0.1% SDS) containing 2 µg/mL protease inhibitors (protease inhibitor cocktail, Cat No: 4693116001; Roche, Germany) and 0.1% phosphatase inhibitor (Phosphatase Inhibitor Cocktail II; Sigma-Aldrich,USA). Supernatants were collected and their protein concentrations were determined using a BCA protein assay kit (Pierce Biotechnology, Rockford, IL, USA). Aliquots of the lysates (each containing 40 mg of protein) were boiled for 5 min and electrophoresed on a 10% SDS–polyacrylamide gel. The resolved proteins were then transferred to PVDF membranes (Millipore, Billerica, MA, USA). Membranes were blocked by incubation in 5% bovine serum albumin at room temperature for 2 h and were then incubated with primary antibody for overnight at 4°C. The primary antibodies were as follows: anti-NDRG2 (Abnova, Taiwan, China), MMP-2, MMP-9 (Santa Cruz Biotechnology, Santa Cruz, CA, USA), phospho-ERK1/2, total-ERK1/2, phospho-p38/MAPK, total-p38/MAPK, phospho-JNK, and total-JNK (Cell Signaling, Bedford, MA, USA). The membranes were then incubated with the appropriate alkaline phosphatase-conjugated secondary antibody (Santa Cruz Biotechnology, CA, USA) for 1 h. Antibody binding was finally detected using an enhanced chemiluminescence Western blot detection kit (Pierce Biotechnology, Rockford, IL, USA).

### Establishment of the animal tumor model

BALB/C athymic nude mice (male, 6 weeks of age) from the Laboratory Animal Research Center of the Fourth Military Medical University (Xi'an, China) were used in compliance with the regulations of the Animal Ethics Committee of the Fourth Military Medical University of the People's Liberation Army. Resuspended HepG2 cells (5×10^6^ cells in 200 µl) were infected separately with either the shRNA-control or shRNA-NDRG2 was injected into the hind legs of the mice. Each experimental group contained 5 mice. After 2 weeks of implantation, mice in the heat-treated groups were subjected to a 45°C water bath for 30 min. Four weeks later, the mice were sacrificed and their primary tumors were removed for further histological examination. All the experimental procedures were conducted in accordance with the Detailed Rules for the Administration of Animal Experiments for Medical Research Purposes issued by the Ministry of Health of China and received ethical approval by the Animal Experiment Administration Committee of the Fourth Military Medical University. All efforts were made to minimize the animals' suffering and to reduce the number of animals used.

### Regional hyperthermia treatment in tumor-bearing mice

Tumors were heated by immersing the tumor-bearing leg in a thermostat-controlled waterbath (YGM Instrument, type DZKW-D-1, Beijing, China). The tumor-bearing leg was pulled down using a sinker, and the tumor was immersed at least 10 mm below the water surface. The temperature of water bath was set at 45°C for 30 min. The temperature at the center of the tumor nodule and the rectal temperatures were measured during the heat treatment with a thermocouple (Physitemp Instruments, type IT-18, USA). The mice were anaesthetized with an i.p. injection of pentobarbital sodium at a dose of 60 mg/kg before administering HT. To reduce systemic heating, the nude mice were cooled using a fan during treatment to prevent whole body HT [9].

### Pathological analysis

Formalin-fixed, paraffin-embedded tumor sections were deparaffinized in xylene, followed by treatment with a graded series of alcohol and staining with hematoxylin-eosin (H&E). For immunohistochemistry, antigen retrieval for paraffin-embedded tissues was performed with sodium citrate, after which the samples were placed in boiling water for 20 min. Endogenous peroxidase was blocked by incubating the sections in 3% hydrogen peroxide in methanol for 10 min. The samples were incubated with rabbit polyclonal antibodies to MMP-2 and MMP-9 (Santa Cruz Biotechnology, Santa Cruz, USA) or PBS (negative control) at 4°C overnight. The samples were then incubated for 30 min with the appropriate dilution of the secondary antibody (ZSGB Biotechnology, Beijing, China), followed by incubation with the HRP-linked streptavidin-biotin complex in a humidified chamber for 10 min at RT. Positive reactions were visualized by incubating the slides with DAB (ZSGB Biotechnology, Beijing, China) for 5 min. The sections were then counterstained with hematoxylin for 15 sec, dehydrated and cleared and observed under a photomicroscope (Olympus BX51, Tokyo, Japan).

### Apoptosis analysis

The cells were collected at the indicated times, washed twice with PBS and incubated in the dark for 15 min with binding buffer [10 mM HEPES/NaOH (pH 7.4), 140 mM NaCl and 2.5 mM CaCl_2_], Annexin V-FITC (200 mg/ml; BD Pharmingen, San Diego, CA, USA) and propidium iodide (PI, 1 mg/ml; Sigma-Aldrich, USA). The fluorescence of Annexin V-FITC and PI were measured using FCM (flow cytometry, Epics Elite flow cytometer; Coulter, Miami, FL, USA). The data were analyzed using Cell Quest software.

### Statistical analysis

All experiments were repeated at least three times. Results are shown as the mean ± SD. The data were analyzed with the SPSS 13.0 software package, and statistical comparisons between groups were made using a one-way ANOVA followed by Student's *t*-test. *P*<0.05 was considered statistically significant.

## Results

### Inhibition of HCC invasion by HT is accompanied by NDRG2 upregulation

HT has been found to successfully inhibit the invasiveness of various cancer cells. Here, we examined the anti-invasive effect of HT on HepG2 and Huh7 cells by subjecting them to water baths at different temperatures (37°C, 39°C, 41°C, 43°C and 45°C) for 30 min. Matrigel invasion assays were performed to evaluate the effect of HT on metastatic activity. As shown in Fig. 1A, the invasiveness of HepG2 and Huh7 cells was not affected by heat treatment at temperatures of 37°C–43°C. Compared with the control group (37°C), heat treatment at 45°C reduced the percentage of invaded cells by 65.4% in HepG2 and 68.7% in Huh7 cells, respectively. There was no statistically significant difference in the percentage of invaded cells between HepG2 and Huh7 cells. To further confirm the anti-invasion effect of HT, we examined the expression of MMP-2 and MMP-9 in both HCC cell lines. As shown in Fig. 1B, the expression of MMP-2 and MMP-9 was significantly reduced by HT at 45°C. In addition, Western blot showed that the expression of NDRG2 was increased by heat shock at 45°C in both HepG2 and Huh7 cells, which was negatively correlated with the down-regulation of MMP-2 and MMP-9. These finding suggest that NDRG2 is induced by heat shock at 45°C and associated with inhibitory effect of HT (45°C) on HCC cells. Therefore, all experiments described below were performed at a heat shock temperature of 45°C in HepG2 cells, which is the most common cellular model for human liver tumors.

**Figure 1:** HT retards the invasion of HCC with up-regulation of NDRG2. (A) HepG2 and Huh7 cells were exposed to different temperatures (37°C, 39°C, 41°C, 43°C and 45°C) for 30 min. Matrigel invasion assays were performed after 24 h of heat treatment in order to evaluate the effect of HT on invasiveness. Cell invasion is shown in phase contrast images and graphical representations. Invasion was assessed by counting cells in five microscopic fields per well at 400×magnification. The data are representative of triplicate experiments and calculated as the means ± SD. The invasion rate of cells at 37°C was defined as 100%, and *P<0.05 indicates the degree of statistical significance as compared to cells at 37°C. (B) Expression levels of NDRG2, MMP-2 and MMP-9 in heat-treated HepG2 and Huh7 cells were determined by Western blot after 24 h of heat treatment at different temperatures (37°C, 39°C, 41°C, 43°C and 45°C) for 30 min. Tubulin was used as the internal loading control.

### Anti-invasion effect of HT is enhanced in NDRG2-overexpressing HCC cells

To elucidate whether NDRG2 is associated with the anti-invasion effects of HT, we established HepG2 cell lines that constitutively expressed NDRG2 protein by lentiviral infection (Fig. 2A, 2B). The overexpression of NDRG2 enhanced the inhibition of invasion in HepG2 cells exposed to HT, which is consistent with results reported previously. In NDRG2 overexpressing cells, heat shock at 45°C significantly reduced the invasive potential of the cells (Fig. 2C) compared with HepG2 cells treated by HT alone. These results indicate that NDRG2 strengthens the anti-invasive effect of HT. We next detected the expression of MMP-2 and MMP-9. Western blot revealed that the expression of MMP-2 and MMP-9 was decreased in NDRG2 overexpressing HepG2 cells and that the expression was even lower after the cells were treated by HT (45°C). These data indicate that NDRG2 might enhance the anti-invasion effect of HT by inhibiting the expression of MMP-2 and MMP-9 (Fig. 2D).

**Figure 2:** NDRG2 overexpression enhances the anti-invasion effect of HT in HCC cells. (A) Expression level of NDRG2 in Control, Cherry (transfected with overexpression control plasmid), and NDRG2 (transfected with NDRG2 overexpression plasmid) cells. (B) NDRG2 expression level in Cherry or NDRG2 cells was determined by Western blot after HT at 45°C for 30 min. (C) The anti-invasive effect of HT was studied in Cherry or NDRG2 cells after HT at 45°C for 30 min. Cell invasion is depicted in the phase contrast images and the graphical representation. Invasion was assessed by counting invasive cells in five microscopic fields per well at 400×magnification. The data are representative of triplicate experiments and were calculated as the means ± SD. The invasion rate of Cherry-37°C cells was defined as 100%. *P<0.05 or **P<0.01 indicatesthe degree of statistical significance compared to Cherry-37°C cells. (D) Expression levels of MMP-2 and MMP-9 in 45°C heat-treated Cherry or NDRG2 cells were assessed by Western blot analysis. Tubulin was used as the internal loading control.

### Down-regulation of NDRG2 attenuates the inhibitory effects of HT on invasion of HCC cells in vivo

To confirm the role of NDRG2 on the invasive capability of heat-treated HCC cells in vivo, we further examined the anti-invasion potential of NDRG2 in HCC-implanted mice. We first established stable NDRG2-deficient HepG2 clones by infecting cells with lentivirus-mediated NDRG2-specific shRNA (shNDRG2-HepG2). The Scramble shRNA sequence was used as a negative control (Scramble-HepG2). As shown in Fig. 3A, the NDRG2-specific shRNA decreased the expression of NDRG2 significantly compared with the Scramble shRNA. NDRG2-deficient HepG2 cells were injected into nude mice and treated as described in the Materials and Methods. H&E staining of histological sections from the mouse xenograft model revealed that HT significantly suppresses the invasion ability of HepG2 cells. As shown in Fig. 3B, malignant tumors slightly invaded into nearby tissues in HT-treated mouse model. In contrast, the suppression of NDRG2 facilitated the invasion of tumor nodules and reversed the anti-invasive effect of HT in HepG2 cells, which was accompanied by a significant destruction of the muscle layer. The expression of both MMP-2 and MMP-9 was also detected in tissue sections, and a representative immunohistochemical staining is presented in Fig. 3C. Consistent with the H&E staining results, we found that down-regulation of NDRG2 alleviated the repression of MMP-2 and MMP-9 expression by HT. These results imply that NDRG2 is involved in the HT-caused inhibition of invasion via the suppression of MMP-2 and MMP-9 expression.

**Figure 3:** Down-regulation of NDRG2 affects the invasiveness of heat-treated HCC cells in vivo. (A) Expression level of NDRG2 in Scramble-HepG2 (transfected with silencing expression control plasmid) and shNDRG2-HepG2 (transfected with NDRG2 silencing plasmid) cells. HepG2 cells were transfected separately with the Scramble or shNDRG2 and then individually injected into the hind legs of the mice. After two weeks of implantation, mice in the heat-treated groups were subjected to a 45°C water bath for 30 min. Each experimental group contained 5 mice. Four weeks later, mice were sacrificed, and primary tumors were removed for histological examination. (B) Representative H&E staining of histological sections revealed histological destruction in each group. Arrows point to invasion areas. Stars mark the locations of muscle. (C) Immunohistochemistry showed expression levels of NDRG2, MMP-2 and MMP-9 in the tumor tissues of each group. Bar = 30 µm (magnification 400×).

### ERK1/2 signaling isreduced in NDRG2-overexpressing cells

Because NDRG2 was responsive to HT, we evaluated the role of NDRG2 in the anti-invasion effect of HT. The overexpression of NDRG2 has been found to inhibit the malignant potential of breast cancer cells in a MAPK-dependent manner. Therefore, we investigated the effect of NDRG2 on the downstream activation of the MAPKs signaling pathway by detecting phosphorylated p38MAPK, extracellular signal regulated kinase1/2 (ERK1/2), and c-Jun NH_2_-terminal kinase (JNK), which were induced by HT. The JNK and ERK1/2 pathways showed high intrinsic basal activation. Neither HT nor NDRG2 overexpression further enhanced JNK activation. On the other hand, the phosphorylation of ERK1/2 increased up to 1.25-fold within 2 h, rapidly declined to the basal level 4 h after heat shock treatment, and then reduced to even lower levels. Moreover, the overexpression of NDRG2 abrogated the intrinsic and HT-induced activation of the ERK1/2 pathway (Fig. 4). HT was found to increase the activation of p38MAPK in a time-dependent manner, whereas the phosphorylation level of p38MAPK remained unchanged in NDRG2-overexpressing cells. These findings indicate that ERK1/2 activation may be selectively inhibited by NDRG2 expression in HepG2 cells.

**Figure 4:** NDRG2 inhibits HT-induced ERK1/2 activation in HCC cells. Cherry (transfected with over expression control plasmid) and NDRG2 (transfected with NDRG2 expression plasmid) cells were subjected to a 45°C water bath for 30 min and then incubated at 37°C for the indicated periods of time. The cells were lysed and levels of ERK1/2, JNK, and p38MAPK were detected by Western blot. Levels of ERK1/2, p38MAPK and JNK phosphorylated proteins at the indicated time points after heat treatment were detected by Western blot and quantitated by measuring band intensities. The values of the fold activations were normalized to the total ERK1/2, p38MAPK or JNK values. The data are representative of three independent experiments and were calculated as the means ± SD. *P<0.05 indicates degrees of statistical significance as compared to Cherry cells. Tubulin served as the loading control.

### NDRG2 mediates the anti-invasion effect of HT via inhibition of the ERK1/2 signaling pathway

To further confirm the role of NDRG2 on ERK1/2 activation, lentivirally infected short-hairpin RNA was employed to down-regulate endogenous NDRG2 expression in HepG2 cells. NDRG2-deficient cells were treated with the ERK1/2 inhibitor PD98059, the p38MAPK inhibitor SB203580 or the JNK inhibitor SP600125, respectively. As shown in Fig. 5A and 5B, silencing NDRG2 expression significantly increased the invasion ability of heat-shocked cells. In addition, PD98059 treatment significantly enhanced the anti-invasive effect of HT and decrease MMP-2/MMP-9 expression in NDRG2-deficient HepG2 cells. In contrast, no changes were observed in SB203580 and SP600125 treated cells. Therefore, our results suggest that ERK1/2 pathway inhibition, but not p38MAPK or JNK pathway inhibition, is responsible for the decreased invasiveness of NDRG2 knockdown HepG2 cells.

**Figure 5:** NDRG2 mediates the anti-invasion effect of HT via the inhibition of ERK1/2 activation. shNDRG2-HepG2 (transfected with NDRG2 silencing plasmid) cells were pre-incubated with 10 µmol/ml PD98059, 10 µmol/ml SB203580 or 50 µmol/ml SP600125 for 30 min before heat treatment at 45°C for 30 min. (A) Cell invasion is represented graphically. The data are representative of triplicate experiments and were calculated as the means±SD. *P<0.05 indicates the degree of statistical significance. (B)MMP-2 and MMP-9 expression levels were determined by Western blot. Tubulin served as the loading control.

### NDRG2 synergizes with HT to inhibit the invasiveness of HCC cells and decrease spontaneous necrosis

HT leads to cell death by either apoptosis or necrosis depending on temperature [26]. Apoptosis, which is a naturally occurring cause of cellular death, often provides beneficial effects to the organism. In contrast, necrosis is almost always detrimental and can be fatal. We examined the type of cell death induced by HT treatment at different temperatures using double staining with Annexin V and PI. HepG2 cells treated at 45°C showed a significantly higher rate of cell apoptosis, compared with those treated at 43°C. Simultaneously, HT at 45°C caused a massive increase in the number of necrotic cells in comparison with cells treated at 43°C (Fig. 6A). Intriguingly, we found that the combination of NDRG2 expression and HT at 43°C resulted in increased apoptosis and reduced necrosis compared with HT at 45°C. Although heat shock at 43°C and NDRG2 expression each induced apoptosis to a certain degree, the effect of their combination exceeded the mere sum of the effect of each treatment alone, thus indicating a synergistic effect. Moreover, the capacity of heat shock and/or NDRG2 expression to affect the invasion of HepG2 cells was assessed. The cells treated at 45°C showed a significantly lower percentage of invaded cells (64.3%) compared with those treated at 43°C (81.5%). The combined treatment of heat shock at 43°C and NDRG2 expression decreased the expression of MMP-2/MMP-9 and reduced the invaded cell percentage by 65.2%. Simultaneously, exposure to the combination of HT at 43°C and NDRG2 expression resulted in less necrosis and reduced the invasiveness of HepG2 cells.

**Figure 6:** NDRG2 enhances the efficacy of HT. (A) The effect of HT on necrosis and apoptosis was studied in Cherry (transfected with over expression control plasmid) or NDRG2 (transfected with NDRG2 expression plasmid) cells after heat treatment at 43°C or 45°C for 30 min. Apoptosis was measured through FACS analysis of PI- or Annexin V-stained cells. Column data analysis of intact cells (Annexin V−, PI−), early apoptotic (Annexin V+, PI−) and late apoptotic/necrotic cells (Annexin V−/+, PI+) for each cell group. *P<0.05 indicates the degree of statistical significance compared to the Cherry-37°C group; **^#^** *P*<0.05 indicates the degree of statistical significance as compared to the Cherry-45°C group. (B)The anti-invasive effect of HT was studied in Cherry or NDRG2 cells after HT at 43°C or 45°C for 30 min. Cell invasion is depicted in the phase contrast images and the graphical representation. Invasion was assessed by counting cells in five microscopic fields per well at 400×magnification. The data are representative of triplicate experiments and were calculated as the means ± SD. The invasion rate of Cherry-37°C cells was defined as 100%. *P<0.05 indicates the degree of statistical significance as compared to Cherry-37°C cells. (C) Expression levels of MMP-2 and MMP-9 in 43°C or 45°C heat-treated Cherry or NDRG2 cells were assessed by Western blot. Tubulin was used as the internal loading control.

## Discussion

As a strong adjuvant treatment, HT has been extensively investigated for its propensity to induce apoptosis and alter the metastatic character of tumor cells. Here, our results revealed that HT at 45°C effectively inhibited the invasive capacity of HCC cells, which was accompanied by the decreased expression of MMP-2 and MMP-9. Further mechanistic investigation demonstrated that the NDRG2-mediated suppression of the ERK1/2 pathway accounted for the decreased invasiveness observed in HepG2 cells treated by HT. Moreover, our results suggest that the constitutive expression of NDRG2 optimized the therapeutic effect of HT by enhancing HT's anti-invasive effects and by decreasing spontaneous necrosisin HepG2 cells.

As a member of the NDRG family, the NDRG2 gene has been shown to be intimately involved in carcinogenesis and cancer progression. In addition, accumulating evidence has shown that the expression of human NDRG2 can be induced by a number of cell stress conditions. For instance, Wang et al. demonstrated that NDRG2 expression is significantly up-regulated by hypoxia or hypoxia-mimetic agents in several tumor cell lines [23]. Another previous study showed that NDRG2 expression is highly responsive to different stress conditions in skeletal muscle [25]. Moreover, the increased expression of NDRG2 was observed during Adriamycin (ADR)-mediated DNA damage response [27]. In accord with these results, we determined that NDRG2 was up-regulated by HT-induced heat stress at 45°C in HCC cells (Fig. 1B and 2B). Therefore, our results together with previous reports support the idea that NDRG2 is stress responsive gene.

In contrast to the similar changes of NDRG2 expression, the biological effect of NDRG2 on tumor cell behaviour appeared paradoxical under different stress. In A549 cells exposed to hypoxic conditions, the ectopic expression of NDRG2 enhanced hypoxia-induced apoptosis. This phenomenon was confirmed by the observation that NDRG2, as a p53-inducible gene, is implicated in the p53-mediated apoptosis pathway in response to DNA damage [27]. Thus, in the above studies, NDRG2 appears to act as a stress-responsive gene in order to facilitate cell death. Contrary to these findings, NDRG2 was demonstrated to be involved in the AKT-mediated protection of β cells against lipotoxicity-induced apoptosis [28]. Moreover, NDRG2 contributes to the hypoxia-induced radio-resistance of Hela cells and the increased chemoresistance of Hela cells to cisplatin [24], [29]. Herein, our data showed that the constitutive expression of NDRG2 enhanced HT-induced apoptosis in HepG2 cells. However, the overexpression of NDRG2 alone did not result in cell apoptosis directly (Fig. 6A), and more important, we found that NDRG2 could potentiate the anti-invasive effect of HT (Fig. 1B, 2C and 2D). The down-regulation of NDRG2 by shRNA attenuated the inhibitory effects of HT on invasion in the nude mouse xenograft model (Fig. 3). We suspect that the alterations of cell responses induced by NDRG2 are complex and depend on the intensity or the type of stress. Another possible explanation is that NDRG2 has different effects on tumor malignancy in a cell context-dependent manner. Further investigations should be conducted to test this hypothesis.

NDRG2 has been reported to be a candidate suppressor of tumor metastasis based on a number of studies. Shon et al. reported that NDRG2 overexpression inhibited the metastatic potential of breast cancer cells through the BMP-4 mediated suppression of MMP-9 activation [21]. Moreover, a previous study showed that NDRG2 suppresses the metastatic potential of HT1080 human fibrosarcoma and B16F10 murine melanoma cells both in vitro and in vivo [30]. Recently, Kim et al. reported that the high expression level of NDRG2 is inversely correlated with tumor invasion depth and Dukes' stage of colon adenocarcinoma [31]. Very recently, NDRG2 expression was found to be down-regulated in gallbladder carcinoma, and the expression level was found to be closely correlated with deeper invasion depth and the TNM stage of the patients. Here, our data showed that the introduction of NDRG2 into HepG2 cells significantly suppressed the expression of MMP-2/MMP-9 and reduced the invasion of cells (Fig. 2C and 2D). These results are consistent with previous findings that NDRG2 plays important roles in suppressing tumor metastasis in HCC [17], [32], [33]. HT at 45°C was found to inhibit HCC invasion, which was accompanied by the upregulation of NDRG2. We speculated that a possible mechanism for the anti-invasion effect of HT is that up-regulated NDRG2, at least in part, contributes to decreased levels of MMPs, thereby resulting in the suppression of cell invasion.

Increasingly more studies have reported that MAPKs seemto play a pivotal role in tumor invasion andmetastasis [34], [35], [36]. Heat exposure, a kind of stress, is associated with the activation of the MAPK family [37], [38], [39]. Our data showed that HT did not alter the activation of JNK (Fig. 4), and a similar result was observed in MDA-MB-231 cells [40]. In addition, we observed that HT inhibited the activation of ERK1/2 and increased the phosphorylation of p38MAPK. More important, overexpression of NDRG2 abrogated the activation of the ERK1/2 pathway, whereas the activation of p38MAPK remained unchanged in NDRG2 overexpressing cells (Fig. 4). The signaling events involved in the heat shock-induced expression of MMPs and decreased invasion were then investigated in HT-treated HepG2 cells infected with shNDRG2. The inhibition of the ERK1/2 pathway using the specific inhibitor PD98059 reduced invasion in HT-treated NDRG2-deficient cells completely. However, the JNK inhibitor SP600125, and the P38MAPK inhibitor SB203580, only partly reversed the decreased cell invasion and expression of MMPs (Fig. 5). These data suggest that ERK1/2 pathway inhibition, but not p38MAPK or JNK pathway inhibition, is responsible for the decreased invasiveness of NDRG2-deficient HepG2 cells, which is consistent with the findings that NDRG2 antagonizes growth factor production via the selective inhibition of ERK1/2 activation in macrophages [41]. In our previous study, p38MAPK phosphorylation was increased by NDRG2 in HepG2 cells [42], which is not consistent with the unchanged p38MAPK activation observed in the present study. We speculate that the phosphorylation of p38MAPK was increased by HT to such a high level that NDRG2 cannot enhance it anymore.

Metastasis is the most frequent cause of death in patients with advanced liver cancer, and it still poses a challenge to the development of successful cancer therapeutics [43]. HT has recently been applied as a technique for raising the temperature locally to treat tumors. In general, the effect of HT has been shown to be markedly enhanced at temperatures above 43°C, whereas heat results in an independent cytotoxic effect on cultured cells in vitro at this temperature. The cytotoxicity of HT was clearly enhanced as the temperature increased. Xie et al. found that higher temperature HT at 45°C strengthened the anti-invasion effects when compared to lower temperature HT in MCF-7 cells, whereas the cytotoxicity of HT also increased [12]. A similar result was also demonstrated in our study. HepG2 cells treated at 45°C significantly attenuated invasiveness compared with those treated at 43°C, whereas the number of necrotic cells increased (Fig. 6A). The HT at 42°C–43°C was able to kill tumor cells and prevented normal cells from being destroyed. Thermal differences between tumor cells and normal cells disappear in temperatures above 45°C. Both tumor cells and normal cells are committed to necrosis under these circumstances [44]. Necrosis physiologically affects groups of contiguous normal cells and results in phagocytosis by macrophages and a significant inflammatory immune response. Thus, to optimize therapies and avoid or minimize side effects, the overexpression of NDRG2 combined with lower temperature HT at 43°C was used to treat HepG2 cells. As expected, HT at 43°C and NDRG2 appeared to concomitantly suppress invasiveness and decrease the necrosis of HepG2 cells. Because HT>43°C cannot be realistically achieved in a clinical setting, the constitutive expression of NDRG2 combined with HT at 43°C could be a promising approach for the treatment of HCC.

In summary, the present study demonstrates that NDRG2 can be upregulated by HT (45°C)-induced heat stress and that it enhances the anti-invasion effect of HT on HCC cells. Further mechanistic investigation revealed that HT-induced NDRG2 is able to suppress activity of ERK1/2 signaling pathway, which is mainly responsible for the attenuated invasiveness in HepG2. Finally, the synergistic cooperation of 43°C HT and NDRG2 effectively reduced cytotoxicity and promote the anti-invasion effects of HT at 45°C. Understanding the molecular mechanisms involved in HT may have valuable implications for developing optimized HT therapies for NDRG2-deficient cancers.
